The article "Optical Resolution Photoacoustic Microscopy Imaging in the Detection of Early Oral Cancer under Image Reconstruction Algorithm" was published in 2022. Journal: Comput Math Methods Med.

# Optical Resolution Photoacoustic Microscopy Imaging in the Detection of Early Oral Cancer under Image Reconstruction Algorithm

**DOI:** 10.1155/2022/6077748

**Published:** 2022-06-17

**Authors:** Liyuan Zhang, Xiaopeng Wang

**Affiliations:** Department of Oral and Maxillofacial Surgery, Qilu Medical College of Shandong University (Qingdao), Qingdao, 266035 Shandong, China

## Abstract

This research was intended to explore the application value of photoacoustic imaging technology based on image intelligent iterative reconstruction algorithm in the detection and diagnosis of early oral cancer. An iterative algorithm model was constructed and systematically analyzed. The algorithm was used to debug the detection of B-scan images on the diameter of the imaging area. The results showed that the sensitivity of line-focused ultrasound detector was 86.72% and the specificity was 80.79%, while the sensitivity of the flat-field ultrasound detector was 63.15% and the specificity was 71.79%. The photoacoustic microscopy imaging technology can clearly observe the rich capillary network on human lips. A part of the vascular network at the depth of 100 *μ*m, 500 *μ*m, and 1000 *μ*m grew out of the reticular capillaries and extended out of the loop-like capillaries, and the diameter gradually expanded. The imaging experiment of the sublingual capillary network in the human body showed that loop-like capillaries were observed, but there were some large blood vessels, which corresponded to the densely distributed blood vessel network under the tongue. The morphological changes of loop-like capillaries can be well observed by photoacoustic microscopy. In conclusion, the reconstructed photoacoustic microscopy imaging technology can realize high-resolution imaging of human oral capillaries and observe the morphological changes of loop-like capillaries, which had a certain application value for the early detection of oral cancer.

## 1. Introduction

The definition of cancer in medicine is a malignant tumor originating from epithelial tissue. As a common malignant tumor, cancer is usually considered to be all malignant tumors [1]. Oral cancer is a general term for malignant tumors that occur in the oral cavity and is a common malignant tumor in the head and neck of the human body. Globally, oral cancer has become a growing health problem [2]. From the perspective of epidemiology and clinicopathology, “oral cancer” can be divided into three types: oral cancer, lip cancer, and oropharyngeal cancer [3]. Oral cancer and oropharyngeal cancer together constitute the top ten most common cancers in the world, with a combined annual incidence of about 500,000 people [4]. Early stage oral cancer usually has no obvious identifiable symptoms, which is not only difficult for patients to detect but also difficult for doctors to detect early stage oral cancer lesions through routine oral examinations, so it cannot be effectively controlled in the early stage of cancer [5]. In addition, the public lacks sufficient awareness of the risk of oral cancer, and many patients often delay for a long time to seek expert consultation after they have symptoms of suspected oral cancer, missing the best treatment time [6]. Due to the lack of effective treatments for cancer, preventive strategies for early detection and early treatment have become the key to reducing cancer mortality [7].

The article "Optical Resolution Photoacoustic Microscopy Imaging in the Detection of Early Oral Cancer under Image Reconstruction Algorithm" was published in 2022. Journal: Comput Math Methods Med.

Since cancer cells are malignant proliferating cells that are not regulated by normal physiological mechanisms, cancerous tissues must be different from normal body tissues in various parameters such as tissue density, hardness, water content, and blood oxygen saturation [8, 9]. The current medical imaging methods reflect these differences as images to determine the location, type, benign, and malignant of tumors and other information to achieve early cancer screening [10]. At present, the detection methods for oral cancer or oral lesions in clinical medical treatment mainly include routine oral examination, narrow-band imaging technology, ultrasonic imaging technology, X-ray photography, and magnetic resonance imaging (MRI) technology [11]. In view of the above shortcomings of these imaging methods and the various requirements of early oral cancer detection, recently photoacoustic imaging technology has gradually developed into a method that can meet the requirements of early cancer screening. It uses the photoacoustic effect as the imaging basis and performs imaging by detecting the ultrasonic waves emitted by biological tissues when absorbing light energy [12]. At the same time of cancer cell metastasis, new blood vessels can be an indicator of early cancer detection, because these new blood vessels contain a large amount of hemoglobin [13], and hemoglobin is the main source of contrast in photoacoustic imaging [14]. This feature makes photoacoustic imaging enjoy great advantages in early cancer detection [15].

Domestic photoacoustic imaging started late, but the development of system miniaturization and integration, the development of key system components, the optimization of theoretical algorithms, and the expansion of application directions have developed rapidly with the joint efforts of researchers [16]. As the most cost-effective way to improve image quality, reconstruction algorithms have always been the focus in the development of photoacoustic imaging. At present, traditional reconstruction algorithms are roughly divided into analytical reconstruction algorithms, iterative reconstruction algorithms, and numerical reconstruction algorithms [17]. In view of the shortcomings of various oral cancer detection techniques currently available [18], this research proposed a new idea based on image reconstruction algorithm to apply optical resolution photoacoustic microscopy imaging technology to oral cancer detection. Combining the high-resolution and high-contrast imaging advantages of optical resolution photoacoustic microscopy on capillaries and the characteristics that early lesions of oral cancer can cause morphological changes in capillaries, it opened up new application areas for the detection of oral cancer and optical resolution photoacoustic microscopy.

The article "Optical Resolution Photoacoustic Microscopy Imaging in the Detection of Early Oral Cancer under Image Reconstruction Algorithm" was published in 2022. Journal: Comput Math Methods Med.

## 2. Materials and Methods

### 2.1. Sample Preparation

After the imaging system was built, it was firstly necessary to test its performance parameters. The phantom is a kind of sample that is very commonly used in photoacoustic imaging to simulate the characteristics of biological tissue, such as light absorption and scattering. It is simple to prepare and easy to control. In this research, carbon fibers, hair strands, phantoms, and mice were used to simulate light scattering and absorption in biological tissues. The phantom was made by mixing and heating agar powder and deionized water. 3 g of agar powder was mixed with 120 mL of deionized water well and heated in a microwave oven until the mixed solution boiled 6-7 times. Then, a magnetic stirrer was adopted to remove the tiny bubbles dissolved in it. When it cooled down to 52°C naturally, 6 mL of skim milk was added and stirred evenly, dropped with 3.26 *μ*m ink using a micro syringe, and then continued stirring until uniform. The mixed solution was maintained at 52°C for about 35 minutes. Finally, it was injected into the mold, and samples such as carbon fiber filaments and hair filaments were added. The optical absorption and scattering coefficients of this phantom were like those of human biological tissue.

In this research, it mainly tested the parameters of the imaging system such as resolution, imaging depth, sensitivity, and uniformity through black tape and phantom experiments. In addition, it adjusted the system hardware and image algorithm through testing.

### 2.2. Principles of Photoacoustic Imaging

According to the research status of photoacoustic imaging, photoacoustic tomography (PAT), photoacoustic microscopy (PAM), photoacoustic endoscopy (PAE), photoacoustic Doppler (PAD), photoacoustic elastography, photoacoustic molecular imaging, and multimodal imaging have been developed with the vigorous development of photoacoustic imaging technology. In this research, the detection and analysis of oral cancer were mainly based on PAT image reconstruction. The physical principle of photoacoustic imaging was the photo-induced ultrasound effect, which referred to the physical process in which the internal characteristics of the tissue change due to the temperature change caused by the radiation heating of the light source under the irradiation of the light source. For process analytical technology (PAT), the imaging process is shown in Figure 1.

The article "Optical Resolution Photoacoustic Microscopy Imaging in the Detection of Early Oral Cancer under Image Reconstruction Algorithm" was published in 2022. Journal: Comput Math Methods Med.

From the analysis of mathematical principles, in the process of biological tissue receiving radiation heating from light source, the process of conduction of heat and expansion pressure to the periphery of the tissue and reaching equilibrium are called thermal relaxation and stress relaxation, respectively. The time required to finally reach thermal equilibrium was defined by the thermal relaxation time *T*_*r*_ and the stress relaxation time *T*_*y*_, respectively, and the equations were as follows:

(1) $$\begin{array}{c} T_{r}=\beta_{c}^{2}\cdot \partial_{r}^{-1},\\ T_{y}=\beta_{c}\cdot \gamma_{y}^{-1}. \end{array}$$

In the above equations, *β*_*c*_ referred to the characteristic length of the thermal inhomogeneity in the radiation area of the light source, *∂*_*r*_^−1^ was the thermal diffusivity (in m^2^/s), and *γ*_*y*_^−1^ represented the propagation speed of ultrasonic waves, which was 1500 m/s in biological tissue. The equation for the relative volume change of the thermal expansion of the biological tissue at the point *α* was as follows:

(2) $$\begin{array}{c} \frac{dF}{F}=sY\left(a\right)+\mu W\left(a\right). \end{array}$$

In equation (2), *s* was the isothermal compressibility coefficient, *μ* referred to the thermal expansion coefficient, and 4 × 10^−4^*S*^−1^ was taken from the soft tissue. *Y*(*a*) and *W*(*a*) represented the variation of the point pressure and temperature, respectively, and *s* was related to the nature of biological tissue itself and can also be calculated by the following equation:

(3) $$\begin{array}{c} S={\left({\rho \gamma }_{y}^{2}Q_{v}\right)}^{-1}Q_{p}. \end{array}$$

In equation (3), *Q*_*p*_ and *Q*_*v*_ represented the isobaric specific heat capacity and the isovolumetric specific heat capacity, respectively, which characterized the endothermic and exothermic capacity of biological tissue, and *ρ* was the density of biological tissue.

Because the laser pulses used in photoacoustic imaging is nanoseconds and the pulse widths is much smaller than *T*_*r*_ and *T*_*y*_, the thermal and stress constraints are satisfied. Therefore, the influence of heat conduction and stress conduction on the heating process of laser radiation can be ignored, which referred to the relative volume change *dF*/*F* ≈ 0. The formula for the initial sound pressure in the tissue was as follows:

(4) $$\begin{array}{c} Y_{0}\left(a\right)=s^{-1}\mu W\left(a\right). \end{array}$$

It was assumed that the photothermal conversion efficiency of the biological tissue *α* point was 100%, and there was a relationship between the laser pulse and the temperature change as shown in the following equation:

(5) $$\begin{array}{c} W\left(a\right)={\left(\rho Q_{v}\right)}^{-1}X_{p}. \end{array}$$

In equation (5), *X*_*p*_ was the light absorption energy density, and the unit was J/m^3^. If equation (5) was substituted into equation (4), the following equation can be obtained:

(6) $$\begin{array}{c} Y_{0}\left(a\right)={\left(\text{s}\rho Q_{v}\right)}^{-1}\mu \cdot X_{p}. \end{array}$$

The Gruneisen coefficient *τ* expressed the efficiency of the deposition of light energy into photoacoustic waves, and *τ* was about 0.11 for water and about 0.25 for soft tissue at room temperature. The equation looked like this:

(7) $$\begin{array}{c} \tau ={\left(\text{s}\rho Q_{v}\right)}^{-1}\mu . \end{array}$$

It could substitute equation (7) into (6) to obtain a simplified expression of the initial sound pressure signal:

(8) $$\begin{array}{c} Y_{0}\left(a\right)=\tau X_{p}. \end{array}$$

According to the theory of ultrasonic generation and propagation, the photoacoustic signal *Y*(*a*, *d*) of the transducer at point *a* at time *d* can be expressed by the following photoacoustic equation:

(9) $$\begin{array}{c} \left(\forall^{2}-\gamma_{y}^{-1}\cdot \frac{\varphi }{\varphi d^{2}}\right)Y\left(a,d\right)=\gamma_{y}^{-1}\mu \cdot \frac{\varphi W\left(a,d\right)}{\varphi d^{2}}. \end{array}$$

For laser pulses satisfying thermal and stress constraints, the thermodynamic equation was as follows:

(10) $$\begin{array}{c} \rho Q_{v}\frac{\varphi W\left(a,d\right)}{\varphi d}=R\left(a,d\right). \end{array}$$

In equation (10), *R*(*a*, *d*) represented the thermal energy absorbed by the biological tissue per unit volume in unit time. After it was substituted into the photoacoustic equation, the below equation could be obtained:

(11) $$\begin{array}{c} \forall^{2}\cdot Y\left(a,d\right)-\gamma_{y}^{-1}\cdot \frac{\varphi }{\varphi d^{2}}\cdot Y\left(a,d\right)={\left(Q_{p}\varphi d\right)}^{-1}\mu \cdot \varphi R\left(a,d\right). \end{array}$$

The time domain solution of the photoacoustic signal can be obtained by combining the Green function, and the equation was as follows:

(12) $$\begin{array}{c} Y\left(a,d\right)={\left(4\pi Q_{p}\right)}^{-1}\mu ∭{\left|a-a^{\prime }\right|}^{-1}\partial a^{\prime }\cdot {\left.\frac{\varphi R\left(a,a^{\prime }\right)}{\varphi d}\right|}_{d^{\prime }=\left|a-a^{\prime }\right|\cdot \gamma_{y}^{-1}}. \end{array}$$

*R*(*a*, *d*) satisfied the below equation:

(13) $$\begin{array}{c} R\left(a,d\right)=X\left(a\right)L\left(d\right)=\theta_{c}G. \end{array}$$

In equation (13), *X*(*a*) represented the distribution of the light absorption coefficient of biological tissue, *L*(*d*) represented the time distribution function of the laser light source, *θ*_*c*_ was the light absorption coefficient, and *G* referred to the luminous flux rate. Equation (12) can be simplified as equation (14) below:

(14) $$\begin{array}{c} Y\left(a,d\right)={\left(4\pi Q_{p}\right)}^{-1}\mu ∭{\left|a-a^{\prime }\right|}^{-1}X\left(a^{\prime }\right)\partial a^{\prime }-L^{\prime }\left(d-\gamma_{y}^{-1}\left|a-a^{\prime }\right|\right). \end{array}$$

In photoacoustic imaging, the photoacoustic signal *Y*(*a*, *d*) collected by each ultrasonic transducer included time and amplitude information. The relative distance between the transducer and the sound source can be determined by calculating the propagation time of the photoacoustic signal in the biological tissue through the time information. The relative magnitude of the biological tissue light absorption coefficient can be determined by the amplitude information. The combination of the two can determine the photoacoustic image of biological tissue.

The article "Optical Resolution Photoacoustic Microscopy Imaging in the Detection of Early Oral Cancer under Image Reconstruction Algorithm" was published in 2022. Journal: Comput Math Methods Med.

### 2.3. Analysis of Image Reconstruction Algorithms

The sound pressure signal collected by the ultrasonic transducer and the image reconstruction algorithm jointly determined the quality of the photoacoustic image. The standard algorithm was used to reconstruct the sparsely sampled signal, which was prone to produce a large number of undersampling artifacts. Compared with hardware conditions, experimental environment, and many random influencing factors, optimizing the performance of the reconstruction algorithm is the cheapest, easiest, and fastest way to improve the effect of photoacoustic images. The iterative reconstruction algorithm firstly inferred the light absorption distribution of biological tissue according to the photoacoustic signal and then compared the theoretical value of the photoacoustic signal with the real value measured by the transducer. A step-by-step approximation method was used to reduce the error, and it should iteratively iterate until the optimal solution was obtained.

The photoacoustic image to be reconstructed can be represented by an *X*-dimensioanl vector *Z* = [*Z*_1_, *Z*_2_, *Z*_3_,⋯,*ZX*_1_,]^*Y*^ and *X* of which referred to the number of pixels of the photoacoustic image. The initial sound pressure signal collected by the ultrasonic transducer can be represented by an *H*-dimensional vector *N* = [*n*_1_, *n*_2_, *n*_3_,⋯,*nH*_1_,]^*Y*^ and N of which represented the number of sampling points of the ultrasonic transducer, which was the product of the number of ultrasonic transducer array elements and the length of each A-Line. At this time, the available equation for iterative reconstruction of photoacoustic image was as follows:

(15) $$\begin{array}{c} \left\{\begin{array}{c} G_{11}z_{1}+G_{12}z_{2}+\cdots +G_{1x}z_{x}=n_{1},\\ G_{21}z_{2}+G_{22}z_{2}+\cdots +G_{2x}z_{x}=n_{2},\\ G_{H1}z_{1}+G_{H2}z_{2}+\cdots +G_{Hx}z_{x}=n_{H}. \end{array}\right. \end{array}$$

In equation (15), *G*_*ab*_(a = 1, 2, ⋯, *H*; *b* = 1, 2, ⋯, *H*) represented the *b*-th pixel *z*_*b*_, and the weight of the projected value of the *a*-th sampling point *n*_*a*_ on the photoacoustic image *Z* was expressed as a matrix as follows:

(16) $$\begin{array}{c} G=\left[\begin{array}{c} G_{11}G_{12}\cdots G_{1X}\\ G_{21}G_{22}\cdots G_{2X}\\ \vdots \\ G_{H1}G_{H2}\cdots G_{HX} \end{array}\right]. \end{array}$$

In view of the fact that in the actual photoacoustic imaging process, the electromagnetic field and mechanical motion could generate noise. Although after signal processing such as filtering, there was still a certain error between the reconstructed image and the actual photoacoustic image. Therefore, the equation can be further expressed as below equation:

(17) $$\begin{array}{c} H=GZ+\text{error}. \end{array}$$

It is the general mathematical formula of the iterative reconstruction algorithm of photoacoustic imaging. Although iterative reconstruction algorithms can reduce artifacts through prior knowledge, the iterative process has a high time cost and cannot meet the needs of real-time imaging, and many iterative reconstruction algorithms have ideal assumptions. Therefore, reconstruction algorithms with faster speed, smaller errors, and fewer constraints are always the research focus of photoacoustic imaging.

The article "Optical Resolution Photoacoustic Microscopy Imaging in the Detection of Early Oral Cancer under Image Reconstruction Algorithm" was published in 2022. Journal: Comput Math Methods Med.

### 2.4. Statistical Methods

The obtained data were analyzed by the SPSS software version 20.0. Specificity and sensitivity analysis of curve resulted from line-focused ultrasound detector and flat-field ultrasound detector. *P* < 0.05 meant that the difference was statistically significant, proving its validity.

## 3. Results

### 3.1. Experimental System Debugging and Test Results

After the above work, the principle and algorithm analysis of PAT optical resolution photoacoustic microscopy had been basically completed. The next step was to debug the system for experiments to verify the feasibility of PAT scanning and the imaging capabilities of the system. The main purpose of the debugging work was to adjust the central axis of the line-focused ultrasound detector to coincide with the central point of the scanning area, and the most critical part was the detection of the B-scan image on the diameter of the imaging area.  Figure 2 shows the result of the system image after debugging and the maximum projection curve of the flat-field ultrasound detector (V319-SU) with the same parameters.

As shown in Figure 2, the response of the line-focused ultrasound detector within the focal area was significantly more uniform than that of the flat-field ultrasound detector, and the signal-to-noise ratio (SNR) was also higher than that of the flat-field ultrasound detector. The sensitivity of the line-focused ultrasound detector was 86.72%, and the specificity was 80.79%; the sensitivity and specificity of the flat-field ultrasound detector were 63.15% and 71.79%, respectively, and there was a significant difference between the two.

After the debugging work was completed, the sizes of the carbon fiber filaments and the hair filaments were measured, respectively, to check the accuracy of the imaging results, as shown in Figure 3.

As shown in Figure 3, the size of the carbon fiber filament was 11 *μ*m, while the actual size was 8.2 *μ*m. The reason for this difference was that the spot size of the scanning lens used in the imaging process was 9.9 *μ*m, which could not distinguish the target object with a size smaller than 9.9 *μ*m.

To verify the imaging ability of the PAT system on biological tissues, the isolated mice were imaged, and the results were shown in Figure 4.

The capillaries of the mice can be clearly seen in the image. As shown in Figure 4, PAT scanning was indeed able to obtain high-resolution and high-contrast images of the target object due to the absence of relative motion during the entire imaging process. Therefore, there was no aliasing or misalignment in the image.

### 3.2. Human Trial Results

To show the clinical feasibility of photoacoustic microscopy in oral vascular imaging, the tongue and lips of 3 female volunteers were imaged. Before the imaging of each volunteer, the plastic wrap was replaced on the imaging end face and disinfect it with alcohol to ensure the cleanliness and personal hygiene of the imaging system. During the imaging process of the system, there was no relative movement between the imaging end face and the target object, the scanning speed was fast, and the system can approach the target object in an inverted manner. Therefore, the imaging experiment of human oral cavity with this system would be very simple and easy. Although the system still had a certain volume, it was still feasible to image the human lips and easily placed parts such as under the tongue. To verify the imaging ability of the system to the human oral cavity, the PAT system was used to image the capillaries of human lips. During the experiment, the experimental volunteers only needed to put their lips on the imaging end face of the system and wait for the scan to complete. At present, since the imaging speed of the system was limited by the repetition rate of the laser pulse, the imaging process was still long and requires volunteers to remain motionless for a long time. However, due to the high flexibility of the system, it can approach the volunteer's lips in any posture, thereby reducing the volunteer's discomfort. Therefore, the capillary images of human lips were successfully obtained using a semi-hand-held optical resolution photoacoustic microscopy imaging system. Some of the image results are shown in Figure 5. This was also the first application of photoacoustic imaging technology to image human lips.

The article "Optical Resolution Photoacoustic Microscopy Imaging in the Detection of Early Oral Cancer under Image Reconstruction Algorithm" was published in 2022. Journal: Comput Math Methods Med.

In the results, the rich capillary network on the human lips can be clearly observed; there was an ulcer-like area in the center of the picture, and the capillaries around the ulcer area were obviously different from normal capillaries. In order to further reflect the layers of blood vessels on the oral mucosa, the blood vessel network was intercepted at depths of 100 *μ*m, 500 *μ*m, and 1000 *μ*m in the three-dimensional data of Figure 5, as shown in Figure 6.

Figure 6(a) was the capillary located at a depth of 100 *μ*m, and it showed that the capillaries in this layer were mainly loop-like capillaries, which referred to the capillaries located in the most superficial layer. Because it was a healthy human oral cavity, the distribution of capillary loops was relatively uniform. With the increase of depth, the size of blood vessels gradually increased. At the depth of 500 *μ*m shown in Figure 6(b), capillaries showing a network-like distribution can be observed, and a part of loop-like capillaries that grow and extend from the reticular capillaries can be observed. As shown in Figure 6(c), at a depth of 1 mm, the diameter of the blood vessel has also increased significantly.

In addition to the lips, the sublingual area was also a place where oral cancer lesions are more likely to occur, and it was also easier to place. Therefore, the system was adopted to conduct imaging experiments on the human sublingual capillary network in this work. However, since it was difficult to keep the tongue still during the experiment, the experimental time was shortened, and the imaging range and pixel number of sublingual capillary imaging were reduced to ensure the experimental effect. In sublingual capillary imaging, the diameter of the imaged area was reduced to 5 mm, and the step size was still 10 *μ*m.  Figure 7 shows the imaging results of sublingual blood vessels in some humans.

The article "Optical Resolution Photoacoustic Microscopy Imaging in the Detection of Early Oral Cancer under Image Reconstruction Algorithm" was published in 2022. Journal: Comput Math Methods Med.

In the image results, the difference between the sublingual capillary and the lip capillary can be seen. The loop-like capillaries were not easily observed, but there were some large vessels, which corresponded to the densely distributed vascular network under the tongue. In addition, obvious dislocation can be seen in the image, which was because the repetition frequency of the laser was only 10 kHz, resulting in a slow scanning speed and a long imaging time. During this period of time, it was difficult to keep the sublingual completely still on the imaging end surface, so the image would appear misaligned. Due to the jitter in sublingual blood vessel imaging, a human oral ulcer model that was relatively easy to obtain better image effects was selected for imaging, and the healing process of oral ulcers was dynamically observed. These experimental results above proved that the system can achieve high-resolution imaging of human oral capillaries.

### 3.3. Oral Test Results

After the above experiments, the imaging capability of the system had been confirmed. The system was then applied to image various parts of the interior of the human oral cavity, including the upper lip, gums, and inner cheeks. However, since the oral cavity was difficult to keep still, the number of pixels of the oral image was reduced by 300 × 300 to reduce the influence of oral shaking and shorten the imaging time. The results are shown in Figure 8.

In Figure 8, both larger capillaries at deeper positions and smaller loop-like capillaries extending from these capillaries can be observed, reflecting the distribution of capillaries in mucosal tissue and growth. The denser loop-like capillaries made the deeper main vessels difficult to observe. These loop-like capillaries were widely distributed on mucous membranes throughout the human body. From the images of capillaries in various parts of the human oral cavity, it was found that the mucosa located in different parts had obvious differences in the distribution of blood vessels and the morphology of blood vessels. Whether these differences were related to differences in the function or structure of the mucosa remains to be further demonstrated. In addition, the physiological state of the mucosa was closely related to the distribution and morphological changes of these loop-like capillaries. When mucosal lesions occurred, the morphological changes of these loop-like capillaries were immediately reflected. If the oral mucosa was ulcerated, inflamed, or cancerous, the loop-like capillaries would not only become unevenly distributed but also elongated, bifurcated, and adhered. In severe cases, the loop-like capillaries would be completely disappear. The loop-like capillaries were evenly distributed and point in the same direction, indicating that the oral mucosa was in a relatively healthy state.

The article "Optical Resolution Photoacoustic Microscopy Imaging in the Detection of Early Oral Cancer under Image Reconstruction Algorithm" was published in 2022. Journal: Comput Math Methods Med.

## 4. Discussion

The system of photoacoustic imaging in system composition, reconstruction algorithm, functional imaging, and other aspects is gradually complete, and it has become an important branch in the field of biomedicine. Photoacoustic imaging is currently divided into PAT, PAM, PAE, and PAD according to the difference in laser irradiation method, center frequency, type of ultrasonic transducer, and imaging resolution [19]. The research of photoacoustic imaging first started abroad, and foreign countries are in a leading position in system development and clinical practice. In 2003, Lihong Wang's group used photoacoustic imaging technology to image the blood vessels of mouse brain in vivo and confirmed the potential of photoacoustic imaging by comparing with the results of pathological anatomy. In China, research work on optical resolution photoacoustic microscopy imaging is also being carried out [20]. Professor Xing Da's group once proposed a dual-modality imaging system that combines optical coherence tomography and optical resolution photoacoustic microscopy. Different from the traditional dual-modality imaging system, this system uses weak coherent light in the optical coherence tomography system to detect photoacoustic signals, which gets rid of the limitation of using piezoelectric ceramic ultrasonic detectors to detect photoacoustic signals and improves the sensitivity of the system [21]. In addition to performing conventional optical resolution photoacoustic microscopy imaging experiments, an image processing algorithm can extract parameters such as blood vessel diameter, total blood vessel length, and blood vessel density of the complex capillary network in the image [22].

In this research, the principle of annular array PAT in two-dimensional space was introduced in detail, and the generation, propagation, sampling, and reconstruction process of photoacoustic signal were analyzed and sorted out from the perspective of physical principle and mathematical equations. After comparison on the software and hardware improvement schemes of photoacoustic imaging, the operability of the optimized reconstruction algorithm was clarified, and the general mathematical equations of the iterative reconstruction algorithm were further summarized. To simulate the characteristics of photoacoustic images of real tumor tissues as much as possible, a program was used to generate complex random geometric phantoms with different physical and physiological parameters, and the grayscale images of mouse angiography were imported for simulation. The photoacoustic signal was detected with a line-focused ultrasound detector, while imaging was performed using a unique rotary scanning method. The rotating scanning mechanism can cover a large imaging area with high scanning speed, while eliminating the relative motion between the imaging target and the imaging interface of the system, which is widely present in other optical resolution photoacoustic microscopy imaging systems. Combined with the unique inverted structure of the system, it is very easy to operate when used and can be suitable for clinical applications such as ophthalmology, stomatology, and dermatology.

The article "Optical Resolution Photoacoustic Microscopy Imaging in the Detection of Early Oral Cancer under Image Reconstruction Algorithm" was published in 2022. Journal: Comput Math Methods Med.

To promote the technology as soon as possible and solve the difficult early screening of oral cancer [23], an optical-resolution photoacoustic microscopy imaging system for early detection of oral cancer was proposed based on the imaging reconstruction. Based on PAT image reconstruction, the principles of photoacoustic imaging and iterative reconstruction algorithms were analyzed, a test experiment was designed based on the characteristics of biological tissues, and then, formal experiments were carried out on the phantom and human body. The application scope of the system was expanded based on the image reconstruction from the local detection analysis to the analysis of the human lips, to the analysis of the interior of the oral cavity.

## 5. Conclusion

This research was proposed to a method for applying optical resolution photoacoustic microscopy to the detection of oral cancer based on an image reconstruction algorithm. The results showed that the reconstructed photoacoustic microscopy imaging technique can realize high-resolution imaging of human oral capillaries and observe the morphological changes of loop capillaries, which had certain application value for the early detection of oral cancer. However, any imaging technique also had its limitations, and photoacoustic microscopy imaging was no exception. The main problem faced by optical resolution photoacoustic microscopy was the asymmetry between the axial resolution and the lateral resolution. Since the axial resolution was determined by the bandwidth and center frequency of the ultrasound detector and the lateral resolution was determined by the wavelength of light, the differences were huge, making this technique significantly less resolution in the axial direction. Moreover, since the imaging process was carried out point by point, it was difficult to achieve real-time imaging at the phasing speed.

The article "Optical Resolution Photoacoustic Microscopy Imaging in the Detection of Early Oral Cancer under Image Reconstruction Algorithm" was published in 2022. Journal: Comput Math Methods Med.

## Figures and Tables

**Figure 1:** Schematic diagram of the principle of PAT.

**Figure 2:** Projected distribution diagram of the maximum value of B-scan image: (a) the response of the line-focused ultrasound detector; (b) the response of the flat-field ultrasound detector.

**Figure 3:** Photoacoustic imaging results of carbon fiber filaments and hair filaments using a transmission rotary scanning system: (a) carbon fiber filaments; (b) hair filaments.

**Figure 4:** Photoacoustic microscopic image of mouse ear capillaries.

**Figure 5:** Capillary network image of human lip. The scale in the figure represented 1 mm.

**Figure 6:** Image of capillary network at different depth positions of human lips: (a) lip capillaries located at a depth of 100 *μ*m (uniformly distributed capillary loops can be clearly seen); (b) the lip capillaries at a depth of 500 *μ*m; (c) the lip capillaries at a depth of 1 mm. The scale in the figure represented 1 mm.

**Figure 7:** Partial image of human sublingual capillary network. The scale in the figure represented 1 mm.

**Figure 8:** Photoacoustic microscopy imaging results of capillaries inside the human mouth: (a) the upper lip; (b) the gingiva; (c) the cheek. The scale in the figure represented 1 mm.

## Data Availability

The data used to support the findings of this study are available from the corresponding author upon request.
